The article "Pullulan: a new cytoadhesive for cell-mediated cartilage repair" was published in 2015. Journal: Stem Cell Res Ther.

# Pullulan: a new cytoadhesive for cell-mediated cartilage repair

**DOI:** 10.1186/s13287-015-0011-7

**Published:** 2015-03-19

**Authors:** Sarah E Bulman, Cynthia M Coleman, J Mary Murphy, Nicholas Medcalf, Aideen E Ryan, Frank Barry

**Affiliations:** Regenerative Medicine Institute, National University of Ireland Galway, Biosciences, Dangan, Galway, Ireland; Smith & Nephew, York Science Park, Heslington, York, YO10 5DF UK; School of Mechanical and Manufacturing Engineering, Loughborough University, Leicestershire, LE11 3TU UK

## Abstract

**Introduction:**

Local delivery of mesenchymal stem cells (MSCs) to the acutely injured or osteoarthritic joint retards cartilage destruction. However, in the absence of assistive materials the efficiency of engraftment of MSCs to either intact or fibrillated cartilage is low and localization is further reduced by natural movement of the joint surfaces. It is hypothesised that enhanced engraftment of the delivered MSCs at the cartilage surface will increase their reparative effect and that the application of a bioadhesive to the degraded cartilage surface will provide improved cell retention. Pullulan is a structurally flexible, non-immunogenic exopolysaccharide with wet-stick adhesive properties and has previously been used for drug delivery via the wet surfaces of the buccal cavity. In this study, the adhesive character of pullulan was exploited to enhance MSC retention on the damaged cartilage surface.

**Methods:**

MSCs labeled with PKH26 were applied to pullulan-coated osteoarthritic cartilage explants to measure cell retention. Cytocompatability was assessed by measuring the effects of prolonged exposure to the bioadhesive on MSC viability and proliferation. The surface phenotype of the cells was assessed by flow cytometry and their multipotent nature by measuring osteogenic, adipogenic and chrondrogenic differentiation. Experiments were also carried out to determine expression of the C-type lectin Dectin-2 receptor.

**Results:**

MSCs maintained a stable phenotype following exposure to pullulan in terms of metabolic activity, proliferation, differentiation and surface antigen expression. An increase in osteogenic activity and Dectin-2 receptor expression was seen in MSCs treated with pullulan. Markedly enhanced retention of MSCs was observed in explant culture of osteoarthritic cartilage.

**Conclusions:**

Pullulan is a biocompatible and effective cytoadhesive material for tissue engraftment of MSCs. Prolonged exposure to pullulan has no negative impact on the phenotype, viability and differentiation potential of the cells. Pullulan dramatically improves the retention of MSCs at the fibrillated surface of osteoarthritic articular cartilage. Pullulan causes an upregulation in expression of the Dectin-2 C-type lectin transmembrane complex.

The article "Pullulan: a new cytoadhesive for cell-mediated cartilage repair" was published in 2015. Journal: Stem Cell Res Ther.

## Introduction

Articular chondrocytes maintain healthy cartilage structure with a low turnover of extracellular matrix components [1]. Following injury, chondrocytes initially attempt to regenerate healthy tissue [2] but their capacity to regenerate new cartilage with appropriate structural integrity is limited and generally a fibrous neo-cartilage of poor quality is produced [3,4]. Osteoarthritis (OA) is a common condition leading to severe pain, loss of joint function and poor quality of life and has a very significant economic and societal burden. There are no treatment modalities available today which either retard or reverse joint degeneration in OA. There is an urgent clinical need for new regenerative therapies for OA and cell replacement therapy presents a promising option. Autologous chondrocyte implantation (ACI), used clinically to treat acute cartilage injury, fails to produce hyaline cartilage, creates harvest site morbidity and has limitations in terms of chondrocyte potential in older patients [5,6]. The effectiveness of this strategy has been limited because of the poor quality of the regenerated tissue, the impact associated with morbidity of the harvested cell donor site and the complex nature of the surgical procedures.

Mesenchymal stem cells (MSCs) represent an attractive chondro-therapeutic because, when implanted *in vivo*, adult bone marrow-derived MSCs have the potential to differentiate into chondrocytes, thus providing an opportunity for the regeneration of articular cartilage [7,8]. In addition, MSCs have demonstrated therapeutic properties, such as the release of immunomodulatory factors and cell chemoattractants, suggesting an indirect effect by enriching the repair environment [9]. In a goat model of traumatic OA local delivery of MSCs to the articular joint slowed the progression of cartilage degradation. However MSCs *in vivo* did not engraft to either intact or fibrillated cartilage in these treated joints [10-12].

There are several ways in which cellular retention may be increased at the cartilage surface [13]. Increasing the cell dose is an option but, due to the limited sources of progenitor cells and costs of harvesting and expansion, this may not be economically attractive [14-16]. Furthermore, the use of biomaterial scaffolds may not lead to improvements in either retention or viability [17-19]. Several approaches have been described to enhance cell retention at a particular tissue. Peptides and antibodies have been used to direct cells to target sites of repair [20,21] and nanomaterials and microcarriers also have potential to enhance cell retention with the added capacity to influence cell behavior [22-25]. However, there is limited clinical experience of these approaches and questions of biocompatibility, feasibility and toxicity *in viv*o are unaddressed [13].

The article "Pullulan: a new cytoadhesive for cell-mediated cartilage repair" was published in 2015. Journal: Stem Cell Res Ther.

Bioadhesives have been used for bonding soft tissues during surgery, as gap-filling agents in orthopaedic reconstruction and more recently, as drug delivery systems [26,27]. An orthopaedic adhesive must possess adequate strength to hold a tissue bond for a sufficient time, be biocompatible to allow natural regeneration and have a degradation rate comparable to that of neotissue formation [26,28]. Bioadhesive bonding of cells to a tissue surface has been explored using hydrogels and cellular encapsulation [29,30]. A biomaterial hydrogel composed of chondroitin sulfate succinimidyl succinate has been used in a number of applications [31-33], such as the encapsulation and delivery of human MSCs for bone repair [34]. The hydrogel has also been used for the delivery of bone marrow and fusion of meniscus fibrocartilage tissues, demonstrating superior mechanical strength and binding [32,35] and successfully applied in the clinic in combination with microfracture [35].

Independent of the mechanism of therapeutic action, cell retention is likely to be critical for efficacious repair [36]. In this study, it was hypothesised that the application of a bioadhesive to the degraded cartilage surface will increase local cellular retention. The cytoadhesive pullulan was evaluated as an adhesive to enhance MSC adhesion and persistence at the articular cartilage surface. Pullulan is a naturally occurring polysaccharide, forming part of the cell wall of the common yeast-like fungus *Aureobasidium pullulans.* It consists of three glucose units connected by α-1,4 glycosidic bonds (maltotriose) and consecutive maltotriose units connected by α-1,6 glycosidic bonds. It is widely used as films, coatings and thickeners in the food and biomedical industry [37,38]. The high adhesion and film-forming abilities of pullulan have made it suitable as a mucoadhesive and in nanoparticles for drug/gene delivery [38,39].

We have assessed the utility of a pharmaceutical grade pullulan as a potential cellular adhesive in cell-mediated tissue repair strategies. The pullulan used had a weight average molecular weight (MW) of 200,000 and demonstrated the desired properties of an erodible wet stick adhesive. Gradual biodegradation of the adhesive was the preferred medium-term behaviour, since it avoids both the long-term residence time that may prevent cell exposure to the native tissue and the short-term residence time typical of a biodegradable polyester that may hydrolyse too quickly in the mildly acidic environment of the inflamed joint. Since a very high MW material would be expected to reside too long in the synovial joint before being degraded to the point where the bulk could be eluted away, the material was chosen based upon an estimated balance between the need for an adequate residence time and the desired biodegradability within the synovial joint.

The article "Pullulan: a new cytoadhesive for cell-mediated cartilage repair" was published in 2015. Journal: Stem Cell Res Ther.

## Methods

### MSC isolation

MSCs were isolated from the bone marrow of consenting human donors ranging in age from 18 to 35 years using a protocol approved by the Clinical Research Ethical Committee at University College Hospital, Galway. Previously described methods were used to isolate and expand cells in culture by direct plating [11]. Cultures were fed twice weekly with MSC expansion medium: Minimum Essential Medium Alpha (α-MEM; Gibco, Life Technologies, Paisley, UK), 10% selected fetal bovine serum (FBS; Lonza, Slough, UK), 1% penicillin/streptomycin (Sigma, Dorset, UK), 2 mM L-glutamine (Sigma), 1% non-essential amino acids (Sigma) and 5 ng/ml recombinant human fibroblast growth factor 2 (rhFGF-2; Peprotech, London, UK) and subcultured after 80% confluence. Cultures were expanded in monolayer to passage 3. For each subsequent assay, three biologic replicates were used.

### MSC viability and proliferation

MSCs were seeded at a density of 3.125 x 10^3^ cells/cm^2^ in a 96-well assay plate and exposed to 0%, 2% and 5% (w/v) pullulan (Hayashibara International, Hayishbara, Nagase, London, UK) for one, three and seven days. Pullulan was UV sterilised prior to use and dissolved in MSC expansion medium. MTS (3-(4,5-dimethylthiazol-2-yl)-5-(3-carboxymethoxyphenyl)-2-(4-sulfophenyl)-2H-tetrazolium), was applied according to the manufacturer’s instructions (Promega, Southampton, UK) and the culture incubated for two hours at 37°C. Culture media absorbance was evaluated at 490 nm on a Wallac Victor™ 1420 Multilabel Counter spectrophotometer.

MSCs were seeded at a density of 5.8 x 10^3^ cells/cm^2^ and exposed to 0%, 2% and 5% (w/v) pullulan for one, three and seven days. Cells were lysed using 0.1% Triton ×-100 (Sigma), scraped, placed in a microcentrifuge tube and subsequently vortexed to pellet cell debris. The Quant-iT PicoGreen double stranded DNA (dsDNA) assay kit (Molecular Probes, Life Technologies, Paisley, UK) was utilised according to the manufacturer’s protocol. Samples were evaluated on a Wallac Victor™ 1420 Multilabel Counter spectrophotometer.

### MSC flow cytometry

MSCs were pre-incubated in tissue culture flasks with 0%, 2% and 5% (w/v) pullulan for a period of one, three and seven days. After incubation, the cells were trypsinised, resuspended in phosphate buffered saline (PBS) (Sigma) at 5 × 10^5^ cells/ml and incubated with phycoerythrin (PE)-conjugated antibodies, CD44 (Milteny biotech, Surrey, UK), CD90 (Abcam, Cambridge UK), CD73 (Abcam), CD105 (Milteny biotech), and an immunoglobulin G (IgG)-PE isotype control (Milteny biotech) at a 1:10 dilution for 20 minutes at 4°C. Cells were washed twice in PBS to remove unbound antibody and resuspended in serum-free α-MEM for analysis using the ExpressPlus program software on the Guava Cytosoft system (Millipore).

The article "Pullulan: a new cytoadhesive for cell-mediated cartilage repair" was published in 2015. Journal: Stem Cell Res Ther.

### MSC differentiation

Tri-lineage differentiation of MSCs was assessed after exposure to 0%, 2% and 5% (w/v) pullulan in MSC expansion media for two hours. For osteogenic differentiation, MSCs were seeded at 3.2 × 10^3^cells/cm^2^ for 24 hours in expansion medium. Cultures were incubated with osteogenic medium (low glucose (Dulbecco’s) Modified Essential Medium (DMEM; Sigma) with 10% FBS, 1% penicillin/streptomycin (Sigma), 50 μM ascorbic acid 2-phosphate (Sigma), 100 nM dexamethasone (Sigma) and 10 mM β-glycerophosphate (Sigma)). Control cultures were incubated in MSC expansion medium for the duration of the assay. Media was refreshed twice a week for 17 days. To visualise deposited calcium, MSCs were fixed, washed and stained in 2% Alizarin Red S solution (Sigma) and photographed using an Olympus IX71 inverted brightfield microscope and QImaging (Retiga Exi) camera. Quantification of calcium was accomplished using the StanBio quantification kit, according to the manufacturer’s instructions.

For adipogenic differentiation, MSCs were seeded at 2.1 × 10^4^ cells/cm^2^ and grown to confluence, changing expansion medium every three to four days. Once confluent, adipogenesis was induced by adding induction medium to the culture (high glucose DMEM with 10% FBS, 1% penicillin/streptomycin, 1 μM dexamethasone (Sigma), 1.7 μM insulin (Sigma), 200 μM indomethacin (Sigma) and 500 μM isobutyl methylxanthine (Sigma)). MSCs were cultured for three days and the medium changed to maintenance medium (high glucose DMEM with 10% FBS, 1% penicillin/streptomycin and 1.7 μM insulin) for a further three days. Alternating media changes were continued for three cycles and then cultures incubated for a further five to seven days in maintenance medium. Negative control cultures were incubated in MSC expansion medium throughout. Cultures were prepared for lipid vesicle visualisation by washing with PBS and cross-linked in 10% neutral buffered formalin (Sigma). Oil Red O solution (Sigma; 0.3% in 99% isopropanol) was added to the cells for lipid staining and haematoxylin (Sigma) was used as a counter stain. Cell lipid vesicles were visualised and photographed using light microscopy. For quantification, Oil Red O was extracted using 99% isopropanol and absorbance read at 520 nm.

The article "Pullulan: a new cytoadhesive for cell-mediated cartilage repair" was published in 2015. Journal: Stem Cell Res Ther.

MSCs were induced to chondrogenic differentiation through pellet culture (2.5 × 10^5^ cells per pellet) in complete chondrogenic medium (CCM; high glucose DMEM, 100 nM dexamethasone, 173 μM ascorbic acid 2-phosphate, 340 μM L-proline, 1% ITS supplement (R&D Systems, Abingdon, UK), 1 mM sodium pyruvate (Sigma), 1% penicillin/streptomycin (Sigma) and supplemented with 10 ng/ml transforming growth factor beta 3 (TGF-β3; R&D Systems). Four pellets per treatment group were prepared and controls were placed in incomplete chondrogenic medium (ICM; CCM without TGF-β3). The culture medium was refreshed twice a week for 21 days. Pellets were histologically processed by cross-linking in 10% formalin, processed through an automated tissue processor (Leica ASP300S) and embedded in paraffin wax. Pellets were sectioned at a thickness of 5 μm using the Leica RM2235 microtome and rehydrated by passing the slides through a series of Histoclear (National Diagnostics, Fisher Scientific, Leicestershire, UK) and graded ethanols, followed by haematoxylin, 0.02% fast green (Sigma), 1% acetic acid (Fisher Scientific, Leicestershire, UK) and 0.1% Safranin O (Sigma) to visualise sulfated glycosaminoglycans (GAG). Slides were then hydrated, mounted and imaged by light microscopy.

Quantitative assessment of GAG content was conducted by DMMB (1, 9 dimethylmethylene blue; Sigma) analysis. Pellets were digested overnight at 60°C in 25 μg/ml papain (Sigma), dissolved in DMMB dilution buffer (50 mM sodium phosphate, 2 mM N-acetyl cysteine and 2 mM ethylenediaminetetraacetic acid (EDTA), pH 6.5). Samples and chondroitin-6-sulphate standards were prepared in DMMB dilution buffer and exposed to DMMB stock solution (in 100% ethanol, deionised H_2_O, 47 mM NaCl, 40 mM glycine and 11.6 M HCl) for five minutes at room temperature with absorbance was detected at 595 nm. The DNA content of each pellet was quantified using the Quant-iT PicoGreen dsDNA assay kit (Molecular Probes) according to the manufacturer’s protocol to assess the GAG/DNA ratio of each pellet.

### Osteoarthritis cartilage explant culture

Informed consent was given by patients with end-stage OA, undergoing total hip and knee arthroplasty as approved by the Clinical Research Ethical Committee at University College Hospital, Galway. Cartilage biopsies were taken from the articular cartilage surfaces of the hip femoral head and condyle tibial plateau of the knee. Full thickness cartilage explants were created by biopsy punch (1 to 2 mm thick and 2 mm diameter). The explants were placed in α-MEM, containing 10% FBS for 48 hours at 37°C and subsequently placed in ICM for 24 hours.

The article "Pullulan: a new cytoadhesive for cell-mediated cartilage repair" was published in 2015. Journal: Stem Cell Res Ther.

### Explant culture with MSCs and pullulan

MSCs were PKH26 labeled with the PKH26GL cell linker kit following the manufacturer’s instructions (Sigma). Explants were incubated in 0%, 2% and 5% (w/v) pullulan for 10 minutes, after which 0.5 x 10^6^ PKH26 labeled MSCs were incubated with each explant on a rocking plate for 20 minutes. Unbound MSCs were removed by washing with PBS, snap-frozen in optimal cutting temperature compound (OCT) embedding medium (RA Lamb) in liquid nitrogen and cryosectioned at 5 μm using the OTF5000 Bright 5040 microtome cryostat. Sections were coverslipped using Vectashield containing DAPI (Vector Laboratories, Peterborough, UK) and visualised using an Olympus BX51 upright fluorescent microscope (Figure 1).

**Figure 1:** **Pullulan-conditioned cartilage.** Schematic shows the methodology for conditioning cartilage with the bioadhesive pullulan prior to MSC delivery. Cartilage biopsies were taken from the articular cartilage surfaces of the tibial plateau of the knee or hip femoral head. The explant surface was coated for 10 minutes in pullulan, an α-1-4; α-1-6-glucan polysaccharide consisting of maltotriose units **(A)**. Culture expanded PKH26-labelled MSCs were applied to conditioned cartilage explants and incubated on a rocking plate for 20 minutes. Unbound MSCs in suspension were removed by washing in PBS, leaving MSCs bound to cartilage which were fixed and analysed histologically **(B)**. MSC, mesenchymal stem cells.

### Stereological assessment of MSC binding

Quantification of cell adherence was performed on 5 μm cryosections of cell-seeded explants. The optical dissector method was used to estimate the number of cells on the surface of the explant [40,41]. The density estimates are expressed as the number of cells present per square millimetre of explant.

### Flow cytometric analysis of dectin-2

Culture expanded MSCs were pre-incubated with 0%, 2% and 5% (w/v) pullulan in expansion medium for 2, 24 and 48 hours. MSCs were trypsinised and resuspended in PBS with 2% FBS at 0.5 × 10^4^ cells/well in triplicate. Cells were incubated with allophycocyanin (APC)-conjugated Dectin-2/CLEC6A antibody (R&D systems) at a final concentration of 6.25 μg/ml for 30 minutes at 4°C, protected from light. Cells were washed twice in PBS with 2% FBS to remove unbound antibody and resuspended in a final volume of 400 μl of PBS with 2% FBS. Immunostaining signal intensity was analysed with a FACSCanto (BD Biosciences, Oxford, UK) with FlowJo software.

### Statistical analysis

All values were expressed as the mean ± standard deviation of the mean (SD). All datasets were tested for significance using two-way analysis of variance (ANOVA). *Post hoc* analysis (Dunnetts) identified where the difference lay within the groups. For all tests, *P* ≤0.05 was considered statistically significant. Data analysis was performed on Minitab 16.2.2.0.

The article "Pullulan: a new cytoadhesive for cell-mediated cartilage repair" was published in 2015. Journal: Stem Cell Res Ther.

## Results

### MSC viability and proliferation are maintained up to seven days in the presence of pullulan

To assess biocompatibility of pullulan towards MSCs, cells in monolayer were exposed to expansion medium containing 0% 2% and 5% pullulan and viability and proliferation assessed after one, three and seven days. An initial increase in metabolism at day 1 was observed in MSCs cultured in 5% pullulan as compared to 0% controls. An increase in metabolic activity was observed at day 7 for both the pullulan-treated and control groups (Figure 2A). PicoGreen analysis of DNA content revealed an increase in cell number in all cultures between days 1 and 3. Treated cultures demonstrated between day 1 and 3 a higher content as compared to controls. At day 7, DNA content continued to increase in untreated cultures, but showed a significant decrease in the pullulan-treated cultures as compared to untreated cells and day 3 content (Figure 2B). Measurement of the metabolic activity per cell (Figure 2C) indicated a decrease after three days in culture and a recovery at day 7. This was the case with both treated and non-treated cells and is hypothesised to reflect the response of the cells to plating density rather than an effect of the polysaccharide.

**Figure 2:** **MSC viability and proliferation was maintained up to seven days in the presence of pullulan. (A)** MSC metabolic activity was assessed by quantitative formazan production (A490). MSCs were cultured in 0%, 2% and 5% pullulan for one, three and seven days. An increase in metabolism at day 1 was observed in MSCs cultured in 5% pullulan as compared to 0% controls. Metabolic activity was maintained at days 3 and 7 in all cultures, but consistently increased over time with no significant change due to pullulan treatment. **(B)** An increase in MSC DNA concentration as assayed by PicoGreen incorporation was observed in all culture conditions between days 1 and 3, with a significant decrease in DNA concentration of MSCs cultured in 2% pullulan after seven days as compared to controls at the same time point. **(C)** The ratio of metabolic activity normalised to DNA content indicated a non-significant increase in MSC metabolism at day 1 in MSCs exposed to 5% pullulan; however, metabolic activity in all cultures decreased with time, returning to day 1 levels at day 7. Data are presented as the mean ± SD of n = 3 biological replicates generated using triplicate measurements, ** = *P* ≤ 0.01. MSC mesenchymal stem cell; SD, standard deviation.

The article "Pullulan: a new cytoadhesive for cell-mediated cartilage repair" was published in 2015. Journal: Stem Cell Res Ther.

### MSC surface phenotype was conserved after short-term pullulan exposure

Assessment of the MSC surface phenotype after pullulan exposure was performed using flow cytometric analysis of the expression of CD44, CD90, CD73 and CD105. Under all conditions, expression of these markers was maintained at 95% to 100% (Figure 3A-C). There was a slight decline in CD73 and CD105 receptor expression in cells exposed to 5% pullulan for longer periods of time (Figure 3C), but all values were well within the range of expression for MSCs. These data suggested that pullulan did not alter the MSC phenotype [42], at least in terms of canonical surface markers.

**Figure 3:** **MSC surface receptor expression decreased over time in the presence of pullulan.** Assessment of CD44, CD90, CD73 and CD105 receptor expression was made by cytometric flow analysis, after one, three and seven days exposure to increasing concentrations of pullulan. **(A)** There was no significant difference in receptor expression between MSCs incubated in 2% and 5% pullulan as compared to 0% controls after one day. **(B)** There was a decrease in overall receptor surface expression for all groups after three days of culture. A decrease was observed in expression of CD90, CD73 and CD105 for MSCs cultured in 5% pullulan after three days compared to 0% and 2% treated cultures; however, it was not statistically significant. **(C)** A further decrease in CD44, CD90, CD105 and a significant decrease in CD73 receptor expression was noted after seven days of MSC culture in 5% pullulan. Data are presented as the mean ± SD of n = 3 biological replicates generated using triplicate measurements, * = *P* ≤0.05. MSC, mesencgymal stem cells; SD, standard deviation.

### MSCs maintain differentiation potential in the presence of pullulan

The effect of pullulan on the capacity of MSCs to undergo trilineage differentiation was determined. MSCs were differentiated in osteogenic, adipogenic and chondrogenic induction media two hours after incubation in 0%, 2% and 5% pullulan and then assessed histologically (Figure 4). A significant enhancement of osteogenic activity was observed in pullulan-treated cultures by Alizarin red staining for calcium deposits (Figure 4). Oil Red O staining of adipogenically-primed cultures indicated a similar abundance of lipids in the cytoplasm of the cells in all treatment groups (Figure 4). Safranin O staining of chondrogenic pellets showed similar GAG deposition in treated and control groups (Figure 4).

The article "Pullulan: a new cytoadhesive for cell-mediated cartilage repair" was published in 2015. Journal: Stem Cell Res Ther.

**Figure 4:** **MSC differentiation was maintained in the presence of pullulan.** Osteogenesis, demonstrated by alizarin red stain showed increased mineral deposition in 2% and 5% pullulan-treated groups as compared to the 0% control. Oil Red O staining of lipid droplets for adipogenesis showed differentiated MSCs in all pullulan-treated groups. Histological assessment by Safranin-O of MSCs in pellet chondrogenic culture showed GAG deposition in all pullulan-treated groups. GAG, glycosaminoglycans; MSCs, mesenchymal stem cells.

### Pullulan dramatically enhances MSC retention on OA cartilage

The objective of this work was to determine if pullulan could act as a cellular adhesive in cell-mediated repair of fibrillated articular cartilage. To determine this, pullulan was applied to OA cartilage explants prior to delivery of PKH26-labelled MSCs. In uncoated explants, delivered MSCs were retained with low efficiency (Figure 5A). However, pre-treatment with 2% pullulan (Figure 5B) resulted in a dramatic increase in cell attachment and retention. A lesser effect, but still substantial, was seen when the cartilage was treated with a higher concentration of pullulan (Figure 5C). Quantification of an estimate of MSC retention using stereology showed an increase in MSC retention to OA cartilage when MSCs were incubated with 2% (2,876 cells/mm^2^) and 5% (1,491 cells/mm^2^) pullulan pre-coated explants as compared to 0% (145 cells/mm^2^) pullulan controls (Figure 5D).

**Figure 5:** **Pullulan enhanced MSC retention on OA cartilage. (A)** PKH26 labelled MSCs (red) bound to fibrillations on DAPI stained human explanted OA cartilage (blue). MSC retention was increased in **(B)** 2% or **(C)** 5% pullulan coated explants. **(D)** Stereological quantification of MSC retention indicated an increase in cell number on 2% and 5% pullulan coated explants as compared to untreated controls. Magnification bars = 100 μm. DAPI, 4′,6-diamidino-2-phenylindole; MSCs, mesenchymal stem cells; OA, osteoarthritis.

### Dectin-2 expression in MSCs dose dependently increases over time following exposure to pullulan

We sought to specifically determine if the dendritic cell-associated C-type lectin-2, the Dectin-2 receptor, is expressed on MSCs in response to pullulan. Dectin-2 is a family of C-type lectin receptors normally upregulated on immune cells in response to exposure to alpha-glucans of fungal and bacterial origin [43-45]. MSCs were incubated with 0%, 2% and 5% pullulan for 2, 24 and 48 hours and Dectin-2 receptor expression analysed by fluorescence activated cell sorting (FACs) (Figure 6). There was a marked time and dose-dependent increase in Dectin-2 expression on MSCs following exposure to pullulan (Figure 6A-B). Some 10% of untreated cells expressed the receptor and this increased significantly to approximately 60% after 48 hours of exposure to pullulan (Figure 6B). In addition to the increased percentage of Dectin-2-expressing MSCs following exposure to pullulan *in vitro*, the mean fluorescence intensity of Dectin-2-expressing cells significantly increased with increasing doses of pullulan and in a time-dependent manner (Figure 6C).

The article "Pullulan: a new cytoadhesive for cell-mediated cartilage repair" was published in 2015. Journal: Stem Cell Res Ther.

**Figure 6:** **Dectin-2 expression on MSCs was significantly upregulated over time in the presence of pullulan.** Histogram plots for MSCs incubated in the presence of increasing pullulan concentrations at 2, 24 and 48 hours **(A)**. Graphs show curve shifts with increasing Dectin-2 staining of cells, with increasing concentrations of pullulan and length of exposure **(A)**. Bar chart representation of Dectin-2 expression on MSCs over time as a result of pullulan exposure (hours) **(B)**. At all time points of exposure, there was an increase in Dectin-2 expression with increasing concentration of pullulan. After 24 and 48 hours, the increase in Dectin-2 expression was significantly increased in 5% pullulan cultures compared to 0% controls. Data are presented as the mean ± SD of n = 3 biological replicates generated using triplicate measurements, ** = *P* ≤0.01; *** = *P* ≤0.001 **(B)**. The mean fluorescence intensity (MFI) of Dectin-2 expression was calculated for MSCs following exposure to increasing concentrations of pullulan over 48 hours. The results of three independent experiments are shown (n = 3 donors) ± SEM **(C)**. MSCs, mesenchymal stem cells; SD, standard deviation; SEM, standard error of the mean.

## Discussion

Culture-expanded MSCs have a capacity to induce a repair response when delivered intra-articularly to the acutely injured or osteoarthritic joint. The therapeutic mechanism may rely upon the capacity of the cells to differentiate into chondrocytes, their immunomodulatory activity or their release of paracrine repair molecules at the site of injury. Whatever the mechanism of action, it is evident that the efficiency of engraftment of delivered cells at the site of cartilage fibrillation is low. In this study, we assessed the ability of the bioadhesive pullulan to increase cell retention at the degraded cartilage surface. We analysed cellular biocompatibility by assessing viability, proliferation, differentiation, and surface marker expression of MSCs exposed to pullulan. We then assessed the ability of pullulan to act as a cytoadhesive to improve the binding of culture-expanded MSCs to human OA cartilage explants. Finally, an analysis of pullulan-mediated receptor up-regulation was carried out to assess a specific receptor response at the cell surface.

The article "Pullulan: a new cytoadhesive for cell-mediated cartilage repair" was published in 2015. Journal: Stem Cell Res Ther.

Pullulan has potential as a biocompatible cytoadhesive for cellular retention in cell therapy applications. MSCs incubated with pullulan demonstrated maintained metabolic activity and proliferation up to seven days. There was a non-significant increase in metabolic and proliferative activity with pullulan, that was likely due to enzymatic breakdown of the polysaccharide [46,47]. Bae *et al.,* looking at methacrylated pullulan hydrogels for engineering microscale tissues, found that pullulan gels promoted cellular proliferation and aggregation of cells compared to gelatin controls [48]. With the ultimate goal of enhancing cell retention, an initial pullulan-stimulated increase in MSC proliferation and aggregation at the cartilage surface may be favourable for increasing cell numbers retained and matrix repair. Several studies [13,17], have suggested that reduced cellular viability, proliferation and retention may contribute to a lack of efficacy in cell-scaffold cartilage scaffold repair. Therefore, the application of pullulan for stimulating proliferation and retention may be an advancement over current technologies.

Analysis of cell surface markers demonstrated maintenance of expression of the International Society for Cellular Therapy-recommended panel of markers [42] over time. This suggested that the phenotypic nature of MSCs was not negatively altered by exposure to the cytoadhesive. The surface receptors CD44, CD90, CD73 and CD105 may be important mediators of MSC activity [49-58] but that relationship may be tenuous. For example, Endoglin (CD105) is required for endothelial cell proliferation and is currently used as a tool to measure tumour angiogenesis [58]. Similarly, CD73 is expressed in several types of cancer and has been associated with increased glioma cell proliferation [57,59]. Therefore, the maintenance of expression of these markers may or may not indicate a useful phenotype.

Differentiation analysis of MSCs in pullulan-treated cultures demonstrated maintenance of chondrogenic and adipogenic potential and an enhancement of osteogenic potential after pullulan exposure. This increase in osteogenesis potentially relates to the increase in proliferation of MSCs in pullulan-treated cultures and may represent an unfavourable response in the context of cartilage repair. Li *et al*. also described enhanced mineralisation in cell monolayers cultured with high glucose [60]. However, reparative MSCs *in vivo* are more likely to provide paracrine support rather than directly contributing to new tissue formation through differentiation [36]. It would also be interesting to further explore the potential of pullulan for cellular adhesion in the field of bone repair and utilise pullulan’s osteogenic potential for implant integration applications [33].

The article "Pullulan: a new cytoadhesive for cell-mediated cartilage repair" was published in 2015. Journal: Stem Cell Res Ther.

The Dectin-2 receptor, a type II transmembrane protein of the C-type lectin family, is expressed on dendritic cells and macrophages [42]. Here, Dectin-2 was also found expressed on the surface of MSCs, an expression pattern directly relating to pullulan dose and exposure. The function of the Dectin-2 receptor, like Dectin-1 for β-glucans, is to induce intracellular cytokines and reactive oxygen species as a protective mechanism from fungal infection [43]. This response is activated through the receptor binding with the Fc receptor γ [42] upon α-glucan binding, activating spleen tyrosine kinase and mitogen-activated protein kinase signalling pathways, inducing NF-κB activation and production of cytokines such as interleukin (IL)-1β, IL-2, IL-6, IL-10, IL12, IL-17A, IL-23, and TNFα [43,44,61]. MSCs are well documented to express IL-6, which has both supportive anti-inflammatory [62-65] and angiogenic properties [66]. However, IL-6 can be pro-inflammatory depending on environmental context and is documented to be increased in OA synovial fluid [67]. Interestingly, Wong *et al*. developed a pullulan hydrogel for delivery in a mouse ischemic wound model and reported pullulan maintenance of cell viability and antioxidant properties, protecting cells from toxic levels of hydrogen peroxide [68]. Further elucidation of pullulan conditioning within the synovial joint and its effects on MSCs through a possible Dectin-2 receptor mechanism will remain for future analysis.

## Conclusions

Pullulan has demonstrated flexibility and compatibility that can be tailored to a specific therapeutic application. It possesses unique properties, such as regular (1 → 6) linkages that impart structural flexibility and high solubility, allowing pullulan to mimic synthetic polymers, but in a stable, non-harmful composition [69]. In this study we have considered the adhesive application of pullulan and demonstrated its physical use for enhancing MSC retention at the diseased cartilage surface with the intention of increasing MSC therapeutic efficacy. Pullulan demonstrated biocompatibility with MSCs including enhanced proliferation up to seven days, with potential for increasing cell numbers *in loco*. Pullulan positively affected MSC osteogenic differentiation, maintaining adipogenesis and chondrogenesis. The addition of pullulan demonstrated enhanced cell retention at the cartilage surface as hypothesised owing to its chosen physical properties as a wet stick adhesive. Furthermore, Dectin-2 receptor surface expression was identified on MSCs in response to exposure to pullulan, suggesting a mechanism by which the MSC binds pullulan and may respond with environmental conditioning in support of local cartilage repair. Therefore, pullulan is a versatile bioadhesive, able to secure MSCs at the articular cartilage surface in support of creating a local reparative environment.

The article "Pullulan: a new cytoadhesive for cell-mediated cartilage repair" was published in 2015. Journal: Stem Cell Res Ther.

## Abbreviations

ACI: autologous chondrocyte implantation
ANOVA: analysis of variance
APC: allophycocyanin
CCM: complete chondrogenic medium
DAPI: 4′,6-diamidino-2-phenylindole
(D)MEM: (Dulbecco’s) modified essential medium
DMMB: 1, 9 dimethylmethylene blue
dsDNA: double stranded DNA
EDTA: ethylenediaminetetraacetic acid
FACs: fluorescence activated cell sorting
FBS: fetal bovine serum
GAG: glycosaminoglycans
ICM: incomplete chondrogenic medium
IL: interleukin
MSCs: mesenchymal stem cells
MTS: 3-(4,5-dimethylthiazol-2-yl)-5-(3-carboxymethoxyphenyl)-2-(4-sulfophenyl)-2H-tetrazolium
NF-κB: nuclear factor kappa-light-chain-enhancer of activated B cells
OA: osteoarthritis
OCT: optimal cutting temperature
PBS: phosphate-buffered saline
PE: phycoerythrin
rhFGF-2: recombinant human fibroblast growth factor 2
SD: standard deviation
TGF-β3: transforming growth factor beta 3
TNFα: tumor necrosis factor alpha
UV: ultra violet
w/v: weight/volume
α-MEM: minimum essential media alpha
